# Design of Table Tennis Training Competition Knowledge Interaction Platform Integrating Improved Swarm Intelligence Algorithm

**DOI:** 10.1155/2022/2594430

**Published:** 2022-08-01

**Authors:** Deqi Li

**Affiliations:** Department of Physical Education, Zhejiang Yuexiu University of Foreign Languages, Shaoxing, Zhejiang 312000, China

## Abstract

Table tennis is China 's national game and the proudest sport in China's sports field. During the research and technology service work of the Chinese table tennis team for many years, it has accumulated a large amount of valuable data on the analysis of skills and tactics of training and matches, match video, training monitoring, and so on. This paper discusses the relevant theory of swarm intelligence algorithm processing big data on the table tennis training competition knowledge interaction platform system, as well as the technical support of Nginx and Tomcat, and determines the technical basis of the table tennis training competition knowledge interaction platform. Through the establishment of the firefly algorithm model, the resource search ability is enhanced, and the traditional firefly algorithm is improved. From the results of the system performance test, it can be found that the improved swarm intelligence algorithm adopted in this paper improves the global convergence, and the load balancing degree gradually decreases with the increase of time. The improved firefly algorithm shows good performance when the bandwidth is low, and the resource occupancy rate is greatly reduced. When the bandwidth is 20, it is reduced by 12.55%. It solves the shortcomings of long time and low success rate, so as to verify the convenience of the system operation and the power of functions and make the platform more intelligent and efficient.

## 1. Introduction

For more than half a century, the Chinese table tennis team has gone through hardships and struggled tenaciously, winning the world table tennis championship time and time again, creating the miracle of Chinese table tennis, occupying a core position in the hearts of the Chinese. It is the pride of the Chinese. This is an aperiodic exercise based on speed, power and flexibility, and aerobic metabolism. It is an organic combination of skill, physical fitness, and intelligence and is characterized by fast speed, many turns, and great strength. Athletes must possess a wide range of physical qualities, including speed, dexterity and coordination, quick reflexes, and explosiveness. Since the 1950s, researchers have proposed many novel intelligent algorithms. For example, the artificial neural network algorithm that abstracts the human brain neuron network from the perspective of information processing, the ant colony algorithm derived from the behavior of ants searching for food to generate a path, and the particle swarm algorithm that iteratively seeks the optimal solution by imitating a swarm of birds or fish are widely used in processing a deeper study of big data analysis and algorithm theory.

Sports teams and research groups collect vast amounts of data during daily training and competition, including game data, training tracking data, sports injury data, physiological and biochemical tests, technical and tactical analysis, and other types of information. The cloud data center is responsible for transmitting these data, and the efficiency and reliability of data transmission will directly affect the performance of the cloud data center. A data migration strategy is the basic requirement for data migration, and it is also a solid guarantee for a stable and efficient system in the future. A good migration strategy can not only reduce migration costs, but also improve cloud data center maintenance and management. Currently, there is no uniform and efficient way to manage this information. How to make full use of these data to provide a platform for coaches and athletes to acquire knowledge and process information and help athletes improve their training levels and achieve good results in various competitions is a problem that needs to be solved.

The focus of this research is on the construction of an interactive platform for table tennis team practice and competition, integrating data in various formats, such as video, image, file, and chart formats. It can provide a simple and efficient interactive interface for table tennis coaches, athletes, scientific researchers, medical staff, managers, etc., to facilitate their acquisition of relevant information, so that all aspects of training management can be refined and improved, and better services are provided for athletes' training and competition. The platform can manage all kinds of team information in a unified way and provide more scientific and reasonable monitoring, evaluation, and decision-making assistance for coaches and athletes' training and competition, so as to help athletes achieve better results.

## 2. Related Work

As things stand, table tennis can be said to be unsurpassed by any sport in China. An essential factor affecting the system design of table tennis robot for automatic detection of table tennis skill and metrics is the spin condition, path, and bouncing power of table tennis. However, the common prediction algorithms could not cope with the data of time sequence and the corresponding spinning state. Zhang researched the methodology of compensated vague neural network-based trajectory prediction for table tennis technical and tactical index automatic detection. Test results showed that the convergence time of the compensated fuzzy neural network was shortened, the training time was shortened, and the prediction accuracy was improved [1].

Deep mining plays an increasingly important role in the formulation of tactics and rules of sports events. Based on the data mining platform, Choi analyzed the correlation between the dynamic score of table tennis and the game performance. Data mining techniques can extract a superset of information from a variety of data sources and then combine this information, so that some patterns and internal relationships can be found. The results showed that the proportion of score reversals gradually decreased as the table tennis game progressed. This was mainly due to physical and psychological factors. Through the analysis of big data, the imbalance between the total score and the game result was explored. Therefore, athletes should carry out targeted combination exercises to reduce the lack of adaptation in the game [2].

Along with the application of computer large data, sports large scale data profiling offers scientific reference for the improvement of athletes' training mode. Based on big data analysis, Zheng analyzed the significance and usage of mental element coaching for table tennis education. In the actual game, psychological quality has become an important foundation for athletes' ability and skills. The usage of the mental factor training in table tennis should make students pay attention to their own characteristics and exercise mental quality on this basis. At the same time, competitive motivation is the main factor affecting the formation of personal emotional changes. Teachers should help players establish correct table tennis motivation [3].

Yilmaz et al.'s study aimed to investigate the effects of the interactive memory system (TMS) and interactive deck in collaborative computer-supported learning (CSCL) on learners' perception of having a social existence and ability to self-regulate. The perceived social presence and self-regulation skills of students in collaborative groups were compared while constructing knowledge on wiki, blog, podcast, and Facebook platforms during CSCL within the scope of the study. When examining the effect of interactive platforms and TMS on self-regulation in terms of self-regulation skills, it was observed that, despite the significant effect of interactive platforms, the effect of the combination of TMS individually and interactive platforms TMS was not significant [4].

With the development of time, data and video information about table tennis training and competitions are increasing day by day. As is known to all, scientific material selection, scientific training, and scientific management are closely related to the improvement of competitive sports level. The fast evolution of technologies in science needs to push the pace of scientific management of sports, for which some research work on swarm intelligence algorithms has been collected.

Recently, group intelligence-based algorithms have become an emerging area of research. Of these, effective solutions to different complex problems have been found with two superheuristic algorithms that were developed recently, that is, the Cuckoo Search Algorithm (CSA) and the Firefly Algorithm (FA). Bhattacharjee and Sarmah attempted to use them to solve combinatorial problems, especially the 01 Knapsack Problem (KP) and the Multidimensional Knapsack Problem (MKP), while in the improved FA, a variable distance shift of the repair operator based on local search and adversarial learning mechanism was used to verify the effectiveness of the algorithm [5].

Ma et al. discussed the algorithm equity of Particle Swarm Optimization (PSO) and a variety of additional newer SI algorithms. Under certain conditions, the primitive releases of SFLA, GSO, FA, ABC, and GSA were identical to the PSO algorithm. Substantiation indicated that the advanced version of ABC performed best on continuous benchmark functions, while the enhanced versions of SFLA and GSA performed best on combined problems with nesting [6].

Ntouni et al. optimized the inspection and testing procedures of spread-based molecular communicative processes by using weighting and detectors that had suitable power transfer values. For this purpose, they proposed a robust iterative optimization algorithm based on standard particle swarm optimization (PSO) techniques, called accelerated-assisted PSO (a-APSO). They implemented the a-APSO operator to estimate the determiner weighing to minimize the error probability in a closed form representation. The results of the study showed that the margin of error outperformed when using A-APSO weights rather than when using weight values available in the literature or when using weights evaluated by standard PSO algorithms [7].

Mashwani et al. proposed a multi-intelligence algorithm (MSIA) for dealing with bounded constrained functions. The performance of the algorithm was evaluated by using a benchmark function with 30 bounded constraints. The algorithm had good convergence and diversity preservation, approximating promising solutions [8].

To verify the data enhancement results of the characteristic choice alcohol system, which is based on the group smart algorithm, Chen et al. conducted experiments in six classes with similar conditions in the first middle school of the city. The experiments showed that, under the feature selection algorithm, students' academic performance was approximately 30% greater than the other methods of teaching, and the sense of cooperation among students reached 0.8. The contradiction between popularity and improvement was solved, and the problem of differentiation and transformation of late-comers was solved [9].

Gao et al. studied the population smart algorithm for the extraction of spatial facial features and hybrid image element breakdown of hyper-spectral distant images. Firstly, two different spatial spectral feature extraction methods were introduced, then linear and nonlinear spectral hybrid models were studied, and then the end element extraction approach based on hybrid quantum cluster of particle optimization algorithm was investigated. The result of experiments showed that the algorithm improved the population based intelligent algorithm for cluster pixel decomposition. The accuracy of the suggested 3DLBP space spectral features for classification was 94.22%. These swarm intelligence algorithms play a great role in solving multivariate data problems and global optimization, but their practicability is not strong [10]. The above research swarm intelligence algorithm and related content of table tennis are analyzed in detail. It is undeniable that these studies have greatly promoted the development of the corresponding fields. Much can be learned from methodology and data analysis. However, there are relatively few studies on table tennis motion by swarm intelligence algorithms, and it is necessary to fully apply these algorithms to the research in this field. The approaches offer a few points of reference for this study, but because of the brief duration and low sample volume of the associated research, this investigation has not yet gained public acceptance.

## 3. Algorithm and Integration

### 3.1. Knowledge Interaction Platform for Table Tennis Training and Competition

With the vigorous development of modern sports, the data about table tennis training and competitions is increasing rapidly, and it is impossible to comprehensively obtain beneficial experience for coaches and athletes only by manually collecting and analyzing the data of previous competitions. In view of the characteristics of table tennis knowledge interaction platform with complex data volume, many user types, and large number of users, role-based access control (RBAC) has been introduced [11]. Its basic idea is to assign access rights to roles and then assign roles to users, and users can only get appropriate access rights through roles. A user can have multiple roles, and the same role can be assigned to multiple users, so there is a many-to-many relationship between users and roles. Users can dynamically activate the roles they own according to their own needs, so they have all the rights to activate the corresponding roles [12]. In RBAC, a user's authority is granted and revoked by assigning and revoking roles, which makes the user's authority and access logically separated, which greatly simplifies authority management [13].  Figure 1 shows the relationship among users, roles, and permissions in the basic principles of RBAC.

Table tennis knowledge interaction platform is a comprehensive management platform. On the one hand, it needs to manage a large amount of data, and on the other hand, it needs to provide a friendly interface for specific users. Therefore, it is divided into two systems: one is a front-end system presented to coaches, athletes, and researchers in the form of a website, providing various data query, professional analysis, retrieval, management, and other functions [14]. And the other is a data input system that provides various data, providing functions such as input, deletion, and management of various data. The data entry system provides functions such as inserting, deleting, and managing various data. The architecture adopts two modes of browser/server (B/S) and client/server (C/S), leverages the strengths of both architectures to deliver coaching, athletes, and researchers with a simple and friendly interface, and ensures the security of the back-end data input system [15]. This is illustrated in Figure 2.

According to the current situation of national table tennis team training, competition and team management, the platform is divided into 6 subcolumns: athlete database, event database, monitoring database, business learning database, team database, and user management, as shown in Figure 3. The tracking database is the core part of the platform and is divided into 5 subsections of training, fitness, form and function, education, and competition monitoring. By monitoring the technical and tactical training level of athletes in routine training or competition training, it is convenient to understand the development trend of athletes' training level.

The Business Learning Library provides literature, videos, and PPT material for technical and tactical analysis. Table tennis literature is divided into many categories, with distinct themes and various forms, including many game videos provided by major domestic and foreign video organizations such as the International Table Tennis Federation and China Network Television, as well as PPT data on the national table tennis team's skill and strategy analysis of domestic and international players during the tournament. A knowledge search engine and video library about table tennis was established for the first time. The scientific information contained in this module is important for improving the cognitive culture and coaching skills of coaches, as well as the coaching skills and athletic performance of players.

### 3.2. Swarm Intelligence Algorithm

Swarm intelligence originates from the research on the group behavior of social insects represented by ants and bees. Swarm intelligence algorithm is a computing technology that evolves according to group behavior. There are many examples of swarm intelligence in nature, such as bird migration, ant colony foraging, fish gathering, and bacterial growth. These gregarious organisms with low individual intelligence behavior gather in ecosystems and adapt to transforming natural environment. Taking ants as an example, Figure 4 shows the foraging behavior of ants. It can be seen that the ants show amazing intelligent behavior in the process of foraging. A is the ant cave, D is the food source, and EF is the obstacle. As shown in Figure 4(b), after a period of time, the information volume of the path BEC is 1/2 of the BFC. After another period of time, 20 ants go from points B, F, and C to food source D, as shown in Figure 4(c). In the following time, more and more ants will choose BFC, and eventually all ants will select BFC. The closest routes among ant burrows and food sources are found by means of ant colonial optimization.

The behavioral norms that should be followed in the swarm intelligence system include several principles: the principle of adaptability, the principle of neighbors, the principle of response diversity, the principle of quality, and the principle of stability. The principle of stability expresses that a group should not change its behavior every time the environment changes. That is to say, individuals should have the ability to adapt to the environment, and when the external environment changes, they should adjust their behavior as soon as possible; individuals should carry out simple information exchange and transmission; group activities should show diversity. There are quality factors that influence each other.

There is no central control in the swarm intelligence algorithm, so when one or several individuals perform poorly, it will not affect the solution of the problem to the entire group. The advantages of swarm intelligence are one of the major reasons why it has become a research hotspot. It has gradually developed into as one of the top priority research topics in the field of Smart Computing. As the research progresses, more and more swarm intelligence algorithms are proposed and applied to more fields; especially the ant colonies intelligence theory of swarm optimization algorithm, particle swarm optimization algorithm, firefly optimization algorithm, etc. have been successfully applied to many fields.

This paper proposed a method, that is, firefly algorithm of improved bandwidth (IB-FA), based on the Firefly algorithm to solve the data migration problem in the cloud computing environment. The IB-FA algorithm adopts a heuristic location selection and placement strategy for the multiobjective constrained optimization problem to realize the data migration problem. In the firefly algorithm process of IB-FA, each server is used to generate a population in the form of firefly individuals, and an objective function that can describe the resource utilization, migration cost, and network bandwidth in the cloud computing environment is designed as the fitness function of the firefly algorithm process in IB-FA, which is used to calculate the absolute brightness of the individual in the firefly algorithm. An individual with a large absolute brightness value can attract an individual with a small absolute brightness value to move to it, and the convergence of the optimal solution can be achieved by an iterative method. However, in the later stage of the classical firefly algorithm, many individuals with relatively small fitness function values will gather near fireflies with better fitness function values, and the distance between individuals gradually shrinks, so the local search ability is weakened accordingly. In response to this problem, the IB-FA algorithm introduces adaptive inertia weights to avoid individual fireflies falling into local optimum. IB-FA obtains the global best problem, which is the final solution when the iteration counts reach the maximum. The improved firefly algorithm can save the bandwidth of the cloud computing data center, improve the load situation of the data center, and, at the same time, help improve the user experience and better realize the optimal location selection strategy for data migration.

### 3.3. Mathematical Description and Analysis of IB-FA

Construct *p* feasible solutions *x*_1_, *x*_2_, *x*_3_,…, *x*_*p*_ in the solution space to represent *m* target data center nodes to be selected, and then, the parameters involved are as follows: the number of fireflies is *p*, *r*_*ij*_ is the distance between fireflies *i* and *j*, the absorption coefficient is *λ*, the absolute brightness is *I*_*i*_ of firefly *i*, and the attractiveness is *α*_*ij*_.

(1) The initial population *X*^*g*^={*X*_1_^*g*^, *X*_2_^*g*^,…, *X*_*p*_^*g*^} of fireflies is initialized, where *X*_*p*_^*g*^ represents the position of the *i*th firefly in the *g*-th generation, *i* ∈ [1, *m*].
(2) The relationship between the absolute brightness *I*_*i*_ of firefly *i* and the objective function value is established. Usually, the objective function is used to describe the absolute brightness. The better the objective function is, the larger the absolute brightness value is; that is,
  (1) $$\begin{array}{c} I_{i}=h\left(X_{i}^{g}\right). \end{array}$$
*h*(*X*_*i*_^*g*^) is defined as
  (2) $$\begin{array}{c} h\left(X_{i}^{g}\right)={\text{acrDC}}_{i}-\upsilon_{j}^{i}. \end{array}$$
acrDC_*i*_ represents the available resources of the *i*th server, *υ*_*j*_^*i*^ represents the migration cost from server *i* to server *j*, *μ* represents the migration cost per minute, *t*_*j*_^*i*^ represents the time required for migration, and *υ*_*j*_^*i*^ is defined as
  (3) $$\begin{array}{c} \upsilon_{j}^{i}=\mu \times t_{j}^{i}. \end{array}$$
(3) Since the traditional attraction calculation only considers the distance between fireflies and the maximum attraction, it does not take into account the absolute brightness of fireflies, which is inconsistent with the actual situation. The method of attraction *α*_*ij*_ is defined. *α*_*ij*_ is defined with regards to the difference between the two fireflies and the official brilliance of the fireflies. If *I*_*i*_ > *I*_*j*_, then the attraction between two fireflies is defined as
  (4) $$\begin{array}{c} \alpha_{ij}=I_{i}\times \exp\left(-\lambda R_{ij}^{2}\right). \end{array}$$
(4) Update the position of fireflies according to the attraction among fireflies. Firefly *j* is drawn to firefly *i* and travels toward firefly *i*. Then, the equation for updating the position of firefly *j* is defined as

(5) $$\begin{array}{c} X_{j}\left(T+1\right)=\omega X_{j}\left(T\right)+\beta_{ij}\left(X_{i}\left(T\right)-X_{j}\left(T\right)\right)+\beta \left(\text{rand}-\frac{1}{2}\right). \end{array}$$

Among them, *X*_*i*_(*T*) represents the spatial position of firefly *i* in iterations *T*. *β* represents the step factor, which is a constant in [0, 1]. In order to avoid the fireflies oscillating back and forth at or near the local extreme point, an adaptive inertia weight *ω* is added, which decreases linearly with the increase of the number of iterations and the objective function, which is beneficial to local search. So, the definition of *ω* is as follows:

(6) $$\begin{array}{c} \omega \left(T\right)=f\left(X_{i}^{g}\right)\times \exp\left(-T\right). \end{array}$$

### 3.4. Formalization of the IB-FA Algorithm

The problem can be formalized as the problem of migrating *q* pieces of data to *p* servers in a cloud data center. The solution can be represented as an n-dimensional vector, where each element value represents the location of the destination server node of the data to be migrated. Assuming that each server node will dynamically change its state according to the load, the impact of different location migration strategies on the data center network bandwidth is also different. A quad is defined as follows:

(7) $$\begin{array}{c} X=\left\{D_{i},\text{DC},B,\text{BS}\right\}. \end{array}$$

*D*_*i*_ represents the set of *q* data to be migrated in the *i*th server, denoted as

(8) Din,γ=D,i1Di2,…,Diq, i∈1,m.

*γ* indicates the time point, and *D*_*ij*_ indicates the *j* th data to be migrated in the *i*th server. DC represents the set of *p* available server nodes, denoted as

(9) $$\begin{array}{c} \text{DC}\left(m,\gamma \right)=\left\{{\text{DC}}_{1},{\text{DC}}_{2},\ldots ,{\text{DC}}_{p}\right\}. \end{array}$$

*B*(*m*, *γ*) represents the network available bandwidth of *m* servers at *γ* time, denoted as

(10) $$\begin{array}{c} B\left(m,\gamma \right)=\left\{B_{1},B_{2},\ldots ,B_{p}\right\}. \end{array}$$

The primary goal of solving the problem in this paper is to find a set of candidate server locations that maximize performance and minimize migration cost, denoted as

(11) $$\begin{array}{c} \text{BS}\left[D_{ij},{\text{DC}}_{m},\upsilon_{m}^{j},\gamma \right],\;\left(i\neq m\right). \end{array}$$

Then, the location node that saves the most bandwidth in the entire data center is selected. *S* represents the sum of the sizes of *q* data to be migrated, denoted as

(12) $$\begin{array}{c} S=\sum_{i=1}^{q}S\left(D_{ij}\right). \end{array}$$

*T* represents the time required for data transmission, and the calculation formula is defined as

(13) $$\begin{array}{c} T=\frac{S}{\text{Bandwidth}}. \end{array}$$

*η* indicates the bandwidth usage of the current server, defined as

(14) $$\begin{array}{c} \eta =\frac{T_{w}}{T_{w}+\sin\theta T_{b}}\times 100\%. \end{array}$$

Since the execution of the background data of each server is constantly changing, the corresponding execution time is also constantly changing. sin*θ* in formula (14) is used to simulate the variation factor *θ* ∈ (0, *π*) of this background data. It can be seen from formula (14) that if the value of *η* is smaller, the server bandwidth occupancy rate is smaller; then, for the bandwidth of the entire data center, there is more bandwidth that can be used to process other transactions, which is conducive to improving the bandwidth utilization of the entire data center.

Niche is a widespread phenomenon in the evolution theory of nature. Biological individuals usually tend to live in the same environment as individuals similar to themselves. It is precisely because of this that nature is full of vitality. Niche originates from the biological idea of a niche, where organisms of the same species live together to create small habitats that, in turn, allow different types of individuals to inhabit them. Applying this idea to computational science means that data with the same trait will be grouped, and data with different traits will be separated, thereby avoiding large datasets around local optimum points and increasing population diversity. The main goal of a niche algorithm is to establish and maintain a stable, diverse subpopulation that can perform parallel evolutionary searches in different research fields, thus solving the problem of optimizing multiple peaks and targets.

Like other smart algorithms, the standard firefly algorithm tends to converge on perfect sites and mature prematurely, improves the efficiency of stereo mapping by using stereo mapping to obtain initialized firefly populations, and provides a basis for population diversity. It uses random momentum weights to change the position update pattern of individual fireflies, striking a better balance between investigative and useable. The timely implementation of niche technologies can not only eliminate the phenomenon of falling into local extremes, but also increase the diversity of populations. The firefly algorithm suffers from falling into local extremes and reducing population diversity at the end of the iteration, so the advantages of the niche technique are used to offset the shortcomings of the basic firefly algorithm.

In general, the initial distribution of individual firefly positions is random, which can lead to an uneven distribution of firefly positions. Therefore, this chapter introduces a chaotic representation with normal and ergodic features to obtain a chaotic initialized population, which not only prevents the algorithm from falling into local optima, but also increases the diversity of the population. Due to the better sequence homogeneity, the cube representation was chosen. The phases of chaos initialization are as follows:

(1) The first individual is obtained. The first firefly is represented by a randomly generated *D*-dimensional vector, *R*=*r*_1_, *r*_2_,…, *r*_*d*_, where *r*_*i*_ ∈ [−1,1], 1 ≤ *i* ≤ *d*.
(2) The remaining *N* − 1 individuals are obtained. Perform *N* − 1 iterations for each dimension equation of *R*:
  (15) $$\begin{array}{c} r\left(n-1\right)=4r{\left(n\right)}^{3}-3r\left(n\right). \end{array}$$
Among them, −1 ≤ *r*(*n*) ≤ 1,  *n*=0,1,2,….
(3) The chaotic variables are mapped to the solution space with the following formula:

(16) $$\begin{array}{c} x_{id}=O_{d}+\left(1+r_{id}\right)\frac{\left(R_{d}-O_{d}\right)}{2}. \end{array}$$

Among them, *x*_*id*_ represents the *d*th dimension coordinate of the *i*th firefly in the solution space; *O*_*d*_ represents the lower limit of the *d*th dimension of the solution space; *r*_*id*_ represents the *d*th dimension of the *i*th individual obtained by formula (16); *R*_*d*_ represents the upper limit of the *d*th dimension of the solution space.

If an individual is closer to the optimal individual, a smaller weight will be generated, thereby speeding up the convergence; if a larger value is generated, a larger fitness function value will be obtained, which is worse than the optimal value; these weights are eliminated. Likewise, the situation is basically the same when the individual is far from the optimal solution. Therefore, in this paper, random inertia weights are introduced into the position update formula, which is

(17) $$\begin{array}{c} x_{i}\left(t+1\right)=v*x_{i}\left(t\right)+\beta \left(x_{i}\left(t\right)-x_{i}\left(t\right)\right)+\alpha \theta_{i},\\ v=\mu_{\min}+\left(\mu_{\max}-\mu_{\min}\right)\times \text{rand}\left(\right)+\lambda \times \text{rand}n\left(\right) \end{array}$$

*μ*_min_ and *μ*_max_ are the minimum and maximum weights, respectively; rand() are the uniformly spread random numbers in the region [0, 1]. *λ* is the measure of the deviation level between *v* and its mean, which is used to correct the weight error of the obtained values to make the weight change towards the ideal weight because, in general, the error of the experimental results follows a normal distribution. rand*n*() is a normally distributed random number.

At the beginning of the iteration, the basic firefly algorithm performs a global search, and there is no need to introduce the niche technology. When firefly populations are highly aggregated, this is an opportune time to introduce niche technologies. When individuals are grouped, it can be seen that the fitness function values of most individuals are relatively close, so the degree of grouping between individuals should be expressed by defining variables, as shown in

(18) $$\begin{array}{c} \phi^{2}=-{\sum_{i=1}^{p}\left(\frac{f_{i}-f_{\text{avg}}}{f}\right)}^{2}. \end{array}$$

Here, *p* is the number of individuals, *f*_*i*_ is the value of the fitness function for the ith individual, and *f*_avg_ is the current average fitness of the firefly population. There is a sufficiently small threshold *T*; when *ϕ*^2^ < *T*, firefly populations are highly aggregated, which is an appropriate time to introduce niche technology. This in turn leads to the exclusion of unsuitable individuals, thereby maintaining population diversity.

### 3.5. Design of Knowledge Interaction Platform for Table Tennis Training and Competition

The knowledge interaction platform system for table tennis training and competition uses the Java language and adopts the J2EE architecture of JDK1.8. The page development uses the powerful EasyUi framework, and the background is built with the SpringMVC framework. The development tool used in this system is Myeclipse2014 or Myeclipse2010. The software development environment is the software required for the development system and its version requirements. The configuration details are shown in Table 1.

Online interactive system has been relatively stable in technology and is in a high development stage. At the same time of development, it also develops a variety of platform technologies. The online platform architecture that is widely accepted and adopted by various user units is the B/S three-tier architecture, as shown in Figure 5.

From Figure 5, a general online system has three layers: front-end server tier, implementation server tier, and database tier. The front-end server tier is to deliver a web-based interface for users. As a learning portal, the main use method is that users log into the front-end web server with a browser, and the server will provide services to users in the form of web pages. The application server layer is the layer that provides the data server layer operation interface for the front-end server layer. The data server layer is the core of providing data services for the entire system. When a user accesses the online learning system through a personal computer or mobile device and performs various operations, the front-end server layer first parses and decomposes the user's operation and then distributes it to the application server. According to the user request forwarded by the front-end server, the application server layer calls the data server layer for service, obtains the read or write information requested by the user, and feeds back the result to the user. The advantages of establishing an online learning system for users in this way are that a common architecture platform can be used, the technology is relatively mature, and an appropriate content platform can be designed according to their own conditions.

Tomcat is one of the most popular web application servers in the world and is well respected by developers and Java developers. Tomcat servers can be unstable and sometimes fail to run due to heavy network traffic, while Nginx can handle large numbers of requests and large amounts of data consistently and efficiently with low resources.

Nginx is a high-performance HTTP server and reverse proxy, which can manage static resources well on multiple high-load websites, separate dynamic and static pages according to programming rules, and use URL hashing, iphash, polling, etc. to balance the load of internal servers.  Figure 6 shows the dynamic and static architecture of the combination of Tomcat and Nginx. Nginx is placed in front of Tomcat as a reverse proxy, so that Nginx can provide static resources such as pictures, js, css, and html.

## 4. Table Tennis Training Competition Knowledge Interactive Platform Simulation Experiment

The main purpose of system performance testing is to test the load capacity and responsiveness of the network and to check the compatibility of the platform's function with the design requirements. The content of performance testing includes the following:

1. Response speed when many users concurrently have access.
2. Resources of the system in case of concurrent access by a large group of users.
3. Network transmission efficiency and stability during concurrent visits by many users.

Figure 7 shows the convergence curves of the model Firefly algorithm and the improved algorithm. From Figure 7, the improved algorithm has better convergence performance.  Table 2 shows the comparison between the firefly algorithm and the improved firefly algorithm. Based on the performance comparison data in Table 2, it can be concluded that the improved hybrid algorithm has better performance in all aspects and shortens the running time of the algorithm.

To validate the efficiency of the improved Firefly algorithm for target location selection policy load balancing of migrated data during cloud data center operation and to compare the bandwidth usage, data values were collected every two weeks for a testing period of 10 weeks. As shown in Figure 8, as the cloud data center operation time increases, the load balancing degree of the two migration strategies gradually decreases. The improved firefly algorithm reduces the load balancing degree of the firefly algorithm. The firefly policy finds the migration location expeditiously. Though it relieves the pressure of burden on the data location pending migratory data, it does not consider the load capacity of the target location in detail, which results in sometimes good load effect and sometimes bad effect. As the bandwidth gradually increases, the ability to process each service becomes stronger and stronger, and the corresponding bandwidth occupancy rate gradually decreases. The firefly policy has considered the resource occupation of the destination position, and the chosen destination position can achieve improved mobility and ensure smoothness. However, compared with the improved firefly algorithm, the effect is not very ideal. The improved firefly algorithm has a higher bandwidth. When the bandwidth is low, it shows good performance, and the resource occupancy rate is greatly reduced. When the bandwidth is 20, it is reduced by 12.55%. Experiments showed that the improved Firefly migration strategy performed better in terms of bandwidth usage and allowed more available bandwidth to serve additional services to other servers in the data center in the cloud due to less bandwidth usage.

The system performance test findings for this platform are presented in Figure 9.  Table 3 shows the total latency for different number of tasks.

From Figure 9, when the system load reaches 50,000 users, it can still respond normally, fully meeting the performance requirements of the system. The improved firefly algorithm can reduce the total delay of the system to a certain extent under different tasks.

System Function Test: training and game monitoring library is extremely important. From 2018 to 2020, 120 matches between the top 35 men in the world rankings (based on the ranking in April 2020) and 130 matches between the 21 women's athletes were selected. Among them, there are 70 competitions for Chinese men's athletes and 50 competitions for men's athletes from other countries; 55 competitions for Chinese women's athletes and 75 competitions for women's athletes from other countries. The technical effectiveness (TE value) of the one-three-beat, two-four-beat, and stalemate ball in each game is calculated, and the percentile method is used to build a technical performance evaluation model for excellent table tennis players. TE ≥ 70% is excellent, and TE < 30% is bad.

After inspection, the data of the athletes' technical performance TE values are all in a normal distribution. According to the technical performance TE value evaluation method, the evaluation grade standards for the technical performance TE values of outstanding male and female table tennis players have been obtained, as shown in Figure 10.

## 5. Conclusion

Table tennis is one of China's competitive sports advantages. As China's national team, table tennis has reached the peak of the international sports world again and again, leading the healthy and vigorous development of China's sports industry. This paper designs and implements a knowledge exchange platform for the training and competition of the Chinese table tennis team based on the current situation of information system applications in the field of sports and the needs of training and competition and team management of the Chinese table tennis team. Through the swarm intelligence algorithm, the game data, game videos, technical and tactical analysis data, training plans within the team, and other data are managed more efficiently and safely, which is a great saving in human and financial effort and helps the team train and play. In the system performance test, when the system load reached 50,000 users, it could still respond normally, fully meeting the performance requirements of the system. And it built a knowledge search engine and video search database based on table tennis, providing a novel knowledge acquisition channel and a personalized communication environment for coaches, athletes, scientific researchers, medical staff, and managers.

## Figures and Tables

**Figure 1:** RBAC fundamentals.

**Figure 2:** Platform structure design diagram.

**Figure 3:** Functional diagram of table tennis team training and competition knowledge interaction platform.

**Figure 4:** Intelligent behavior of ants during foraging. (a) The two paths selected by A–D. (b) Variation of pheromones in two paths. (c) Final path selection.

**Figure 5:** B/S three-layer structure of a project.

**Figure 6:** Dynamic and static separation architecture of Tomcat combined with Nginx.

**Figure 7:** Concentration curves of the firefly algorithm and the modified firefly algorithm.

**Figure 8:** Load balancing comparison chart and comparison chart in terms of bandwidth usage.

**Figure 9:** System performance test results.

**Figure 10:** Evaluation criteria for TE value of technical performance of outstanding male and female table tennis players.

**Table 1:** Software development environment.

Environment	Configuration requirements	Environment	Configuration requirements
Operating system	Windows 10	Browser	IE9 and above or Firefox, Google
Database server	Sql server 2008 or above	Java development environment	Jude v6.1
Application server	Tomcat 8.0	UML modeling tools	Jude v6.1

**Table 2:** Comparison of the firefly algorithm and the modified firefly algorithm.

Performance indicators	Firefly algorithm	Improved firefly algorithm
Running time	46.31 s	33.52 s
Average value	2.4121*e* − 7	5.3247*e* − 9
Optimal value	3.5214*e* − 7	1.2457*e* − 9
Worst value	6.6485*e* − 6	2.6458*e* − 8

**Table 3:** Total latency under different number of tasks.

Number of tasks	Firefly algorithm of improved bandwidth	Improved firefly algorithm
20	985	976
40	1252	1112
60	1520	1441
80	1630	1530
100	2840	2006
120	3001	2541
140	3060	2733

## Data Availability

The data used to support the findings of this study are available from the author upon request.
